# Analysis of Clinical, Serological, and Imaging Features of Autoimmune Pancreatitis and a Case-Control Study on Prognostic Factors in Response to Hormone Therapy

**DOI:** 10.1155/2022/4829467

**Published:** 2022-07-09

**Authors:** Zhiyong Liu, Kai Zhu, Chuanhui Sun, Yun Shen, Shifang Qu

**Affiliations:** ^1^Department of Rheumatology and Immunology, Wuhan University, Renmin Hospital, Wuhan, China; ^2^Department of Pathology, Changzhi Medical College, Heping Hospital Affiliated to Changzhi Medical College, Changzhi, China; ^3^Department of Geriatrics, The Sixth Hospital of Wuhan, Affiliated Hospital of Jianghan University, Wuhan, China

## Abstract

**Objective:**

The paper aimed to analyze the clinical, serological, and imaging features of autoimmune pancreatitis (AIP) and the prognostic factors affecting hormone therapy.

**Methods:**

A total of 106 patients with AIP enrolled in our hospital from March 2016 to August 2018 were treated with the hormone. The curative effect and recurrence were followed up. The patients were divided into relapse group (*n* = 42) and nonrelapse group (*n* = 64) according to the recurrence within 3 years after initial hormone therapy. The symptoms and signs, laboratory examination, and treatment were compared, and binary logistic regression was employed to explore the risk factors of AIP recurrence.

**Results:**

Among the 106 patients included in this study, there were 78 males and 28 females, with a male-to-female ratio of 3:1. The average age of onset was 56.25 ± 8.87 years; the minimum age was 39 years; and the maximum age was 7 years. The main clinical symptoms were jaundice (67.92%), abdominal pain (48.11%), and abdominal distension (33.96%). In addition, there were symptoms of weight loss, nausea, vomiting, itching, and gray stool. Previous complications included 27.35% diabetes (29/106), 22.64% hypertension (24/106), 35.84% smoking (38/106), and 28.30% alcohol consumption (30/106). The serological characteristics were mainly the increase in serum IgG4 level; 92.45% (98/106) level was higher compared to the upper limit of normal value; the median level was 11.65 g/L; and the highest level was 35.79 g/L. A total of 88.67% (94/106) had an abnormal liver function. The results of imaging examination indicated that 58.49% (62/106) of extrapancreatic organs were involved, of which 46.22% (49/106) were the most common bile duct involvement. All the patients in the group reached a state of remission after hormone treatment. After the disease was relieved, the patients were followed up for 3 years. The recurrence rate was 39.62% (42/106), and the median time of recurrence (month) was 9 (range 2–36). The recurrence rates within 1, 2, and 3 years were 20.75%, 31.13%, and 39.62%, respectively. Among the recurrent patients, 52.38% (22/42) relapsed within 1 year, 78.57% (33/42) within 2 years, and 100.00% (42/42) within 3 years. Multivariate analysis showed that the short duration of glucocorticoid therapy and involvement of extrapancreatic organs were risk factors for relapse after glucocorticoid therapy in patients with type I AIP.

**Conclusion:**

Type 1 AIP is more common in middle-aged and elderly men. The clinical symptoms of jaundice, abdominal pain, and abdominal distension are common, often accompanied by involvement of extrapancreatic organs, of which bile duct involvement is the most common. Type 1 AIP glucocorticoid treatment acceptance and disease remission are better, but the recurrence rate is higher after glucocorticoid treatment. Patients with a short time of glucocorticoid treatment and involvement of extrapancreatic organs may have a higher risk of recurrence.

## 1. Introduction

The concept of autoimmune pancreatitis (AIP) was first put forward by Yoshida et al. in 1995 [1]. The clinical manifestation of AIP is often obstructive jaundice. Its first symptoms were emaciation, fatigue, and abdominal discomfort, and there were diffuse or segmental enlargement of the pancreas, irregular stricture of the pancreatic duct, and other imaging manifestations, and the level of serum immunoglobulin G4 (IgG4) increased [1]. In 2001, Hamano et al. reported elevated serum IgG4 levels and related systemic diseases in Japanese AIP patients, which was an important discovery in the study of IgG4-related diseases (IgCG4-RD) [2]. Since then, with the deepening of the study, the histological and cytological features of AIP have been further recognized, which is characterized by lymphocytic sclerosing pancreatitis (LPSP). The histopathology is characterized by CD4 positive T cells and a large number of IgG4 positive plasma cells infiltration, mainly located around the pancreatic duct, accompanied by pancreatic acinar cell atrophy, interstitial striated fibrosis, and occlusive venous phlebitis, which often lead to stenosis and occlusive fibrosis of the main pancreatic duct [3]. About 60% to 80% of AIP patients demonstrate obstructive jaundice with sclerosing cholangitis (IgG4-associated sclerosing cholangitis, lgG4-sC) and other organs, in which cholangiography features are similar to primary sclerosing cholangitis, pancreatic cancer, or cholangiocarcinoma. In 2006, Kamisawa et al. put forward the concept of systemic sclerosis with fibrosis and massive infiltration of IgG4 positive plasma cells based on multifocal fibrosclerosis, which deepened people's understanding of AIP.

Type 1 AIP is easy to relapse, but the research on predicting the risk of recurrence is very limited [4]. According to international consensus, diffuse enlargement of the pancreas, the persistent high level of IgG4, the slow decrease of IgG4 level, increase in serum IgG4 level after glucocorticoid treatment, and proximal IgG4-associated sclerosing cholangitis may be predictive factors for the recurrence of AIP [5–8]. Some patients relapsed after rituximab treatment, and these patients reappeared with different circulating IgG4 positive plasma cells and indicated enhanced somatic hypermutation, indicating that the pathogenesis of the disease is related to the T-cell-dependent response of immature B cells re-recruited by CD4+T cells, which may drive a self-reactive disease process [9, 10]. In order to identify recurrence as soon as possible, it is recommended that patients who respond to initial treatment be followed up regularly.

Steroids can induce remission in most type I AIP patients (about 90%) [11]. Japanese guidelines and international consensus have recommended steroids as a first-line drug for all active and symptomatic untreated AIP patients unless the patient has contraindications or significant drug side effects [11]. Hormones can correct the abnormal localization of transmembrane conductance regulators in abnormal cystic fibrosis of pancreatic ducts and regenerate atrophic acinar cells in AIP, thereby reducing inflammation and fibrosis and improving endocrine and exocrine functions of the pancreas [10, 11]. Therefore, the short-term prognosis of hormone therapy for AIP is positive. For patients with contraindications to hormone therapy, Corrado et al. found that rituximab, a specific drug for CD20 antigen on the surface of B lymphocytes, can also be employed as a single drug to induce remission of AP [12]. At present, it is commonly employed to treat patients with hormone intolerance and recurrent AIP. Some studies have indicated that maintenance therapy with rituximab (1,000 mg/6 months) can significantly reduce the recurrence rate of AIP. However, the long-term prognosis of type I AIP is still unclear. The purpose of this study was to observe the efficacy and recurrence of hormone therapy in patients with AIP and to explore and analyze the clinical, serological, and imaging features of autoimmune pancreatitis and the prognostic factors affecting the response to hormone therapy.

## 2. Patients and Methods

### 2.1. General Information

A total of 106 patients with type I AIP were treated in our hospital from March 2018 to August 2020. The standards are as follows: (1) the diagnosis of AIP was in accordance with the consensus of diagnostic criteria for type 1 AIP made by the International Association of Pancreatology in 2010 (ICDC) [13]: (1) diffuse pancreatic enlargement with delayed enhancement was grade 1, and pancreatic segmental or focal enlargement with delayed enhancement was grade 2. (2) Pancreatography showed that long or multiple main pancreatic duct stenosis without proximal dilatation was grade 1, and segmental or focal main pancreatic duct stenosis without proximal dilatation was grade 2. (3) the serum 1gG4 level of the patients was > 1.35g. (4) Pancreatic lesions involve other organs. (5) Pancreatic histology has at least three typical manifestations of grade 1. (6) the imaging manifestations of pancreatic or extrapancreatic lesions were relieved or improved within 2 weeks after hormone treatment. Type 1 AIP can be diagnosed with grade 1 imaging criteria plus any one nonimaging standard. If grade 2 imaging findings, more than two nonimaging criteria are needed, or combined with histology or hormone therapy, type 1 AIP can be diagnosed (focal lesions should be excluded from pancreatic cancer). According to the presence or absence of obstructive jaundice, abdominal pain, low back pain, and weight loss, Patients with AIP were divided into symptomatic and asymptomatic patients. All patients were regularly followed up in the outpatient clinic for more than one year. All patients received hormone and drug treatment according to doctor's orders. Patients and their families informed consent to this study. Exclusion criteria: the data were incomplete, or the follow-up time was less than 1 year.

### 2.2. Treatment Scheme

Hormone therapy was given oral prednisone at an initial dose of 30–40 mg/d or 0.6 mg/(kg d) for more than 4 weeks, followed by a reduction of 5–10 mg every 2 months to a maintenance dose of 5 mg/d for more than half a year.

### 2.3. Observation Index

Relevant data were harvested by inpatient and outpatient medical record system, including general information, symptoms, and signs (abdominal pain, abdominal distension, jaundice, itching, ascites, nausea, vomiting, gray stool, and weight loss) and past history (diabetes, hypertension, smoking, and drinking history).

In the early morning, 5 ml from peripheral venous blood of fasting patients was harvested and put into the heparin anticoagulant tube, then left at room temperature for 30 minutes, and then centrifuged at 4,000 r/min speed for 15 minutes, and the serum was separated for serological tests (blood amylase, urine amylase, blood lipase, aspartate aminotransferase, glutamate aminotransferase, alkaline phosphatase, glutamyl transpeptidase, serum albumin, total bilirubin, direct bilirubin, indirect bilirubin, bile acid, serum IgG, serum IgA, serum IgM, serum IgG4, and CA199).

Imaging examination: CT and image analysis were performed using American GE64 spiral CT. Scanning parameters are as follows: tube voltage 120 kV, exposure 200 mAs, layer thickness 5 mm, and matrix 512 × 512. CT enhanced intravenous bolus injection of nonionic contrast agent 70∼90 mL and velocity 5 mL/s. The contents of the CT graphic analysis included the changes in the overall shape of the pancreas (diffuse thickening, enlargement of the head of the pancreas, and reduction of the tail of the pancreas), changes in peripancreatic fat space (clear and blurred), vascular involvement, biliary system changes (biliary obstruction, bile duct thickening, truncated changes, pancreatic duct dilatation, or truncated changes), lymph node enlargement, organ involvement, mass enhancement, and capsule-like enhancement.

### 2.4. Statistical Analysis

SPSS21.0 statistical software was used to evaluate the statistical significance of results. And the measurement data were tested by normal distribution and variance homogeneity analysis to meet the requirements of a normal distribution or approximate normal distribution, presented as $\bar{x}\pm s$. *T*-test was employed to compare the two groups, and the counting data were represented by *n* (%). The *χ*^2^ test was employed to compare the mean of multiple groups. Univariate analysis of variance and univariate and multivariate logistic regression analysis were used to screen the risk factors of recurrence after hormone therapy in patients with type I autoimmune pancreatitis. *P* value <0.05 was considered statistically significant.

## 3. Results

### 3.1. Clinical Manifestation

Among the 106 patients included in this study, there were 78 males and 28 females, with a male-to-female ratio of 3:1. The average age of onset was 56.25 ± 8.87 years old; the minimum age was 39 years old; and the maximum age was 78 years old. The main clinical symptoms were jaundice (67.92%), abdominal pain (48.11%), and abdominal distension (33.96%). In addition, there were symptoms of weight loss, nausea, vomiting, itching, and gray stool. Previous complications included 27.35% diabetes (29/106), 22.64% hypertension (24/106), 35.84% smoking (38/106), and 28.30% alcohol consumption (30/106).

The serological characteristics were mainly the increase in serum IgG4 level; 92.45% (98/106) level was higher than the upper limit of normal value; the median level was 11.65 g/L; and the highest level was 35.79 g/L. A total of 88.67% (94/106) indicated abnormal liver function, which was characterized by the increase of glutamyl transpeptidase (90/106), alkaline phosphatase (87/106, 82.07%), aspartate aminotransferase (80/106, 82.1%), alanine aminotransferase (82/106, 82.1%), and direct bilirubin (81/106, 76.41%), as well as glutamyl transpeptidase (94.91%), alkaline phosphatase (87.07%), aspartate aminotransferase (82 pm), and direct bilirubin (76.41%). In some patients, bile acid and total bilirubin increased, and serum albumin decreased. When patients were tested for immunoglobulin, the increase in serum total IgG levels was more common; the total IgG level increased by 60.37% (64/106); the IgA increased by 3.77% (4/106); and the IgM decreased by 16.98% (18/106), and 61.32% of the patients tested for CA199 were elevated.

The results of imaging examination indicated that 58.49% (62/106) were involved in extrapancreatic organs, of which 46.22% (49/106) were involved in the bile duct, 6.60% (7/106) in salivary glands, 13.21% (14/106) in lymph nodes, 5.66% (6/106) in kidneys, and 2.83% (3/106) in lungs. Among the patients with extrapancreatic organ involvement, single organ involvement accounted for 80.55% (58 × 72); two organs involvement accounted for 22.22% (16/72); and three organs involvement accounted for 4.16% (3/72). The three organs were the bile duct, salivary gland, and lymph node.

### 3.2. Treatment Condition

All the patients in the group reached a state of remission after hormone treatment. After the disease was relieved, the patients were followed up for 3 years. The recurrence rate was 39.62% (42/106), and the median time of recurrence (month) was 9 (range 2–36). The recurrence rates within 1, 2, and 3 years were 20.75%, 31.13%, and 39.62%, respectively. Among the recurrent patients, 52.38% (22/42) relapsed within 1 year, 78.57% (33/42) within 2 years, and 100.00% (42/42) within 3 years. All the results are detailed in Table 1.

### 3.3. Comparison of General Condition and Clinical Symptoms between Recurrent Group and Nonrecurrent Group

According to the recurrence within 3 years after the initial treatment, the patients were divided into two groups: 42 cases in the recurrence group within 3 years and 64 cases without recurrence within 3 years. Through the comparison, it was found that the time of the first hormone treatment between groups was statistically significant (*P* < 0.05). Compared with the nonrecurrent group within 3 years, the proportion of short time of hormone treatment in the recurrent group was relatively higher (*P* < 0.05). There existed no significant difference in sex, age, symptoms, and signs and initial hormone dose (*P* > 0.05). All the results are detailed in Table 2.

### 3.4. Comparison of Serological Indexes between Recurrent Group and Nonrecurrent Group

There existed no significant difference in serological indexes (*P* > 0.05), as indicated in Table 3.

### 3.5. Comparison of Imaging Changes between Recurrent Group and Nonrecurrent Group

Through the comparison between groups, it was found that the involvement of extrapancreatic organs was statistically significant (*P* < 0.05). The proportion of extrapancreatic organ involvement in the recurrent group was relatively higher compared to the nonrecurrent group within 3 years (*P* < 0.05). All the results are detailed in Table 4.

### 3.6. Multivariate Analysis of Recurrence in Patients with Type I AIP after Corticosteroid Therapy

Multivariate analysis indicated that the short time of corticosteroid therapy and involvement of extrapancreatic organs were the risk factors of recurrence in patients with type I AIP after corticosteroid therapy (*P* < 0.05), as indicated in Table 5.

## 4. Discussion

As a local manifestation of IgG4-related autoimmune diseases, type 1 AIP is chronic autoimmune-related pancreatitis, which is significantly different from type 2 AIP in clinical manifestations, serological manifestations, and systemic organ involvement [3, 4]. It is recognized that the elevated level of serological IgG4 is recognized by people, and misdiagnosis occurs because the imaging findings are similar to those of pancreatic and bile duct malignant tumors, but type I AIP has a good response to glucocorticoid therapy, which is contrary to the treatment of malignant tumors, so it is necessary to distinguish them clinically [14]. Type1 AIP is the most common in Asian countries, and its earliest concept was proposed by Japan [4]. In recent years, with the understanding of the disease in China, the research on AIP is gradually increasing.

This study indicated that the average age of onset is 56.25 ± 8.87 years old; the minimum age is 39 years old; the maximum age is 78 years old; and the minimum age is 41 years old [6–8]. The incidence among males is 3 times higher than in females, which is consistent with the results of the study that 90% of patients are over 40 years old and the ratio of male to female is 3–4:1 in South Korea [15]. The clinical manifestations of type 1 AIP are often nonspecific and easy to be confused with other abdominal diseases, such as mild abdominal pain, obstructive jaundice, weight loss, new-onset diabetes, enlarged pancreas, or extrapancreatic lesions. The common clinical symptoms of this study were jaundice (72/106, 67.92%), abdominal pain (51/106, 48.11%), and abdominal distension (36/106, 33.96%). Bile duct involvement is relatively common in a study in the United States. The proportion is about 20% and 50% [16]. In this study, 58.49% (62) of the patients had extrapancreatic organ involvement, of which 46.22% (49/106) bile duct involvement was the most common. More than half of the patients with extrapancreatic organ involvement were related to the characteristics of pancreatic manifestations of type I AIP as IgG4-related diseases, suggesting that the occurrence of type 1 AIP is often accompanied by other IgG4-related diseases, which is consistent with the fact that more than 60% of IgG4-related diseases are involved in foreign studies [17]. In the pancreas, as a gland with two parts of endocrine and exocrine secretion, the occurrence of type 1 AIP may lead to endocrine function damage and islet dysfunction. In this study, 27.35% of the patients were confused with diabetes. A study in Japan found that pathological findings were related to changes in islet cells and ductal cells caused by this disease. About half of people with type 1 AIP develop diabetes [18].

A study in the United States found that 70–80% of patients with type 1 AIP had elevated serum IgG4, but 5% of normal people and 10% of patients with pancreatic cancer also had elevated serum IgG4 [19]. When the serum IgG4 cutoff value is the upper limit of the normal value, the sensitivity and specificity for the diagnosis of IgG4-related diseases are 82.8% and 84.7%, respectively, while when the serum IgG4 cutoff value is 2 times the upper limit of the normal value, the specificity increases to 96.2%, the negative predictive value increases to 97.7%, the sensitivity decreases to 56.9%, and the positive predictive value increases to 44.5% [20]. In this study, the serum IgG4 level was on the high side; 92.45% (980.106) was higher than the upper limit of the normal value; the median level was 11.65 g/L; and the highest level was 35.79 g/L. Although the results were higher compared to those in the United States, they all suggested that the increase in serum IgG4 level was a significant feature of the disease. The serum IgG4 level of more than 2 times the normal limit was also employed as the first-grade evidence of a serological diagnosis in ICDC. Its high specificity suggested that clinicians should highly suspect the diagnosis of IgG4-related diseases when the serum IgG4 level was more than 2 times the normal upper limit and avoid false positive as far as possible. When the level of serum IgG4 is ≥140 mg/dL, the sensitivity and specificity of diagnosing type 1 AIP are high [21]. Considering that the level of serum IgG4 can also be increased in some normal subjects and patients with pancreatic cancer, only relying on the level of serum IgG4 in the diagnosis of AIP may be false positive, especially misdiagnosed as a malignant tumor, which will have a serious impact on treatment. When the increase in serum IgG4 level is less than 2 times the upper limit of the normal value, more attention should be paid to histological and imaging evidence. In this study, the vast majority of patients with abnormal liver function, mainly glutamyl transpeptidase, alkaline phosphatase, aspartate aminotransferase, alanine aminotransferase, and direct bilirubin, increased, and the level of CA199 increased, which is consistent with foreign studies [22].

Glucocorticoid therapy is currently the first choice for the treatment of type 1 AIP [23]. Glucocorticoid therapy can relieve the disease continuously and quickly, with a remission rate of 98% in the Japanese national study and 99.6% in the international AIP multicenter study [24]. In this study, all patients achieved remission after glucocorticoid treatment, which may be related to the small sample size. Its treatment is mainly divided into induced remission, maintenance therapy, and retreatment after recurrence. Hormone therapy is the main treatment in each stage. In terms of dose, prednisolone 0.6 mg/kg/d or prednisone 40 mg/d is generally employed as the initial dose [25]. The initial dose of prednisone in this study is lower compared to other reports. Based on the prednisone dose, the median initial dose of hormone of 30 mg and the maximum initial dose of 40 mg can be considered to increase the initial dose of the hormone when all aspects of the patient's state permit.

It is worth noting that type 1 AIP is prone to recurrence, and most patients can achieve remission in the short term, but the recurrence rate in long-term follow-up is about 30–50% [26]. In this study, the recurrence rate is 39.62% (42/106), and the median time of recurrence (month) is 9 (range 2–36). The recurrence rates within 1, 2, and 3 years were 20.75%, 31.13%, and 39.62%, respectively. Among the patients with recurrence, 52.38% (22/42) recurred within 1 year, 78.57% (33/42) within 2 years, and 100.00% (42/42) within 3 years, which was consistent with the results of other studies [25]. At present, the recurrence rate in different studies is sometimes very different, which may be due to the insufficient sample size due to the low incidence of the disease; the treatment has not reached a unified standard; and the standards for recurrence and remission are different. In this study, the recurrence rates within 1, 2, and 3 years were 20.75%, 31.13%, and 39.62%, respectively. This is similar to the results of a retrospective study of 138 cases of type 1 AIP in South Korea [27]. The recurrence rates within 1, 3, and 5 years were 10.9%, 37.2%, and 44.8%, respectively, but half of the patients in this study relapsed within 1 year. This is much different from the fact that the number of recurrence cases in Korea accounts for 22.7% of the total number of recurrence cases within one year, which may be related to the small number of treatment plans or samples. Among the recurrent patients, 85.7% (18/21) developed within 3 years of follow-up, suggesting that clinicians should pay attention to the treatment of the disease in the early stage of the disease, especially in the first 3 years, and pay attention to close follow-up, so as to detect and deal with the recurrence as early as possible [28]. The overall recurrence rate of the Korean study was 47.8%, which was higher than that of this study, but the median follow-up time was 60 months. The team conducted a similar study with a median follow-up time of 24 months and found that the recurrence rate was 32.4%. In this study, the median time of glucocorticoid treatment was 9 months; the shortest was 2 months; and the longest was 36 months. However, at the 2016 International Pancreatic Society (IAP), experts discussed and considered the international consensus on the treatment of AIP. Type 1 AIP should be treated with glucocorticoid maintenance therapy for more than 3 years. The treatment time of glucocorticoid in this study is significantly lower than that of the international consensus. Although most patients have been treated for more than 1 year and their compliance is fine, there is still a gap compared with the international recommendation of 3 years. Therefore, clinicians should pay attention to disease education.

Studies have indicated that long-term low-dose continuous hormone therapy (more than 3 years) helps reduce the recurrence rate, and the recurrence rate of patients receiving hormone maintenance therapy is half lower than that of patients without maintenance therapy. And low-dose hormone therapy can reduce the risk of severe hormone-related side effects [29]. A retrospective study involving 510 patients in Japan showed that prednisolone 2.5–5 mg maintenance therapy for 3 years can reduce the recurrence rate, and hormonal side effects are prone to occur for more than 5 years. Many studies suggested that 3 years seemed to be a suitable course of glucocorticoid therapy, and it was suggested that the duration of hormone maintenance therapy should be prolonged appropriately. However, other studies have found that even with low-dose cortical maintenance therapy; the recurrence rate is still between 5 and 30%, suggesting that there are other factors affecting the recurrence of type I AIP [30]. Japanese scholars believe that patients with type 1 AIP should use low-dose glucocorticoid for early maintenance therapy, while western scholars only recommend maintenance hormone therapy after recurrence. Compared with hormone therapy, the effects of immunosuppressants, biological agents, and biliary drainage are not satisfactory. It is not recommended to be employed alone in the absence of hormone contraindications, but it can be combined with hormone therapy. Or as a supplementary treatment after recurrence, there are few patients who use the above methods in this study, and they have no effect on the recurrence rate [30].

In recent years, the research on the risk factors related to the recurrence of type 1 AIP has been gradually carried out, but because of the low incidence of the disease and the need for a long follow-up time, the current research generally has the problems of small sample size and short follow-up time, and most of them are retrospective studies, so there are many differences in the long-term prognosis of the disease [31]. A systematic review and meta-analysis found that a large proportion of AIP patients relapsed after successful glucocorticoid induction therapy (33%), especially in patients with type 1 AIP (37%). Maintaining glucocorticoid therapy for more than 1 year can reduce the risk of recurrence [31, 32]. A study found that the recurrence rate of glucocorticoid maintenance therapy for 3 years (23.3%) was significantly lower than that of glucocorticoid treatment for 6 months (57.9%), suggesting that long-term corticosteroid maintenance therapy may reduce the recurrence rate [32]. In this study, the median time of glucocorticoid treatment in the recurrent group within 2 years was 9 months, while that in the nonrecurrent group within 3 years was 36 months. The time of glucocorticoid treatment in the nonrecurrent group was about 2 times longer compared to the nonrecurrent group. It is suggested that while paying attention to the side effects of glucocorticoids, the use of glucocorticoids should be prolonged according to the condition.

A retrospective analysis in Japan suggested that obstructive jaundice may be an important predictor of recurrence, but in this study, there existed no significant difference in obstructive jaundice. A prospective cohort study of IgG4-related diseases conducted at Peking Union Medical College Hospital 76 indicated that elevated serum IgG4 levels may indicate recurrence, while a UK prospective cohort study I84 l indicated that serum IgG4 levels greater than 2 times the upper limit of normal levels could predict the risk of recurrence of IgG4-related diseases, but another study did not support this view [14]. In this study, the median levels of serum IgG4 in the recurrent group and the nonrecurrent group were 15.72 g/L and 16.21 g/L, respectively, and there existed no significant difference. The increase in serum IgG4 level is an obvious characteristic of type 1 AIP. Other studies have found that the persistent high levels of IgG4, the slow decrease of IlgG4 level, the increase in serum IgG4 level after glucocorticoid therapy, and other related factors can predict the recurrence of type 1 AIP, suggesting that it is of great value in the risk of recurrence, and further study is needed. In the future, we can further explore the changes in serum IgG4 levels in the treatment of the disease and carry out prospective research. A retrospective study in France indicates that cholangitis and other organ involvement may be risk factors for recurrence in type 1 AIP; a Japanese study suggests that retroperitoneal fibrosis may be an important risk factor for recurrence; and another study found that bile duct damage is usually a manifestation of disease recurrence, and dilated involvement and poor serum response suggest a higher risk of recurrence. The above studies suggest that the involvement of extrapancreatic organs, especially the bile duct, may be related to the recurrence of type 1 AIP. Univariate binary logistic regression analysis indicated that extrapancreatic organ involvement might be a risk factor for recurrence, but there existed no significant difference in bile duct involvement. In addition, there existed no significant difference in salivary gland involvement, lymph node involvement, lung involvement, and kidney involvement between the two groups (*P* > 0.05). It may be due to the small sample size or the limited source of patients in our hospital. Compared with the nonrecurrence group, the proportion of extrapancreatic organ involvement in the recurrence group was higher compared to the nonrecurrence group within 3 years. In addition, there were no significant differences in age, gender, initial dose of hormones, liver function, CA199, and other symptoms and signs between the groups. For the recurrence of type 1 AIP, it is necessary to conduct regular follow-ups and fully popularize the science of education. Some scholars suggest that imaging examination should be carried out 4 times every 6 months and laboratory examination should be carried out every 3–6 months. For the study of type 1 AIP, expanding the sample size and prolonging the follow-up time will be helpful for further exploration.

Conclusively, type 1 AIP is more common in middle-aged and elderly men. The clinical symptoms of jaundice, abdominal pain, and abdominal distension are common, often accompanied by extrapancreatic organ involvement, of which bile duct involvement is the most common. Type 1 AIP had better glucocorticoid treatment acceptance and disease remission but a higher relapse rate after glucocorticoid treatment. Patients with short-duration glucocorticoid therapy and involvement of extrapancreatic organs may be at higher risk of recurrence.

## 5. Disclosure

Zhiyong Liu and Kai Zhu and share the first authorship.

## Figures and Tables

**Table 1:** The recurrence rate of the patients with AIP.

Follow-up time	The number of recurrences	Recurrence rate (%)

Within 1 year	22	20.75
Within 2 years	33	31.13
Within 3 years	42	39.62

**Table 2:** Comparison of general information and clinical characteristics between the recurrent group and nonrecurrent group (*n* (%), $\bar{x}\pm s$).

Index	*N*	Recurrent group (*n* = 42)	Nonrecurrent group (*n* = 64)	*χ* ^2^/*t*	*P*

Age	106	55.98 ± 9.25	56.13 ± 8.74	0.084	0.932

Gender					
Male	78	30 (38.46)	48 (61.54)	0.166	0.683
Female	28	12 (42.86)	16 (57.14)		

Course of disease (month)	106	4.19 ± 1.65	4.26 ± 1.87	0.197	0.844

BMI (kg/m^2^)	106	25.53 ± 3.17	25.54 ± 4.83	0.011	0.990

Diabetes history					
Yes	29	11 (37.93)	18 (62.07)	0.047	0.827
None	77	31 (40.26)	46 (59.74)		

Jaundice					
Yes	72	30 (41.67)	42 (58.33)	0.392	0.531
None	34	12 (35.29)	22 (64.71)		

Abdominal pain					
Yes	51	22 (43.14)	29 (56.86)	0.507	0.476
None	55	20 (36.36)	35 (63.64)		

The stomach is swollen					
Yes	36	17 (47.22)	19 (52.78)	1.316	0.251
None	70	25 (35.71)	45 (64.29)		

Initial time of hormone therapy (month)	106	9.56 ± 2.53	15.72 ± 3.86	9.127	<0.001

Initial dose of hormone (mg)	106	39.28 ± 6.12	40.75 ± 7.11	1.098	0.274

**Table 3:** Comparison of serological indexes between recurrent group and nonrecurrent group $\left(\bar{x}\pm s\right)$.

Index	*N*	Recurrent group (*n* = 42)	Nonrecurrent group (*n* = 64)	*t*	*P*

IgG4 (g/L)	106	15.72 ± 2.14	16.21 ± 2.56	1.026	0.306
CA199 (IU/ml)	106	44.35 ± 6.53	46.22 ± 4.14	1.805	0.073
Blood amylase (U/L)	106	69.27 ± 11.28	72.16 ± 15.64	1.033	0.303
Urinary amylase (U/L)	106	155.28 ± 16.66	161.85 ± 18.24	1.876	0.063
Blood lipase (U/L)	106	102.27 ± 14.22	99.24 ± 9.54	1.313	0.191
AST (U/L)	106	113.76 ± 18.21	108.33 ± 16.89	1.569	0.119
ALT (U/L)	106	98.34 ± 17.46	103.28 ± 12.74	1.682	0.095
ALP (U/L)	106	313.75 ± 25.27	306.55 ± 26.71	1.386	0.168
ALB (g/L)	106	34.63 ± 5.46	36.59 ± 5.74	1.752	0.082
T-BIL (*μ*mol/L)	106	93.76 ± 7.26	96.13 ± 8.45	1.491	0.138
D-BIL (*μ*mol/L)	106	58.67 ± 8.57	55.89 ± 6.79	1.856	0.066
I-BIL (*μ*mol/L)	106	30.58 ± 4.89	31.28 ± 4.63	0.744	0.458
BA (*μ*mol/L)	106	28.35 ± 5.11	26.88 ± 3.49	1.760	0.081

**Table 4:** Comparison of imaging changes between the recurrent group and nonrecurrent group (*n* (%)).

Index	*N*	Recurrent group (*n* = 42)	Nonrecurrent group (*n* = 64)	*χ* ^2^	*P*

Salivary gland involvement					
Yes	7	3 (42.86)	4 (57.14)	0.032	0.856
None	99	39 (39.39)	60 (60.61)		

Lymph node involvement					
Yes	14	6 (42.86)	8 (57.14)	0.070	0.790
None	92	36 (39.13)	56 (60.87)		

Lung involvement					
Yes	3	1 (33.33)	2 (66.67)	0.051	0.821
None	103	41 (39.81)	62 (60.19)		

Kidney involvement					
Yes	6	2 (33.33)	4 (66.67)	0.105	0.745
None	100	40 (40.00)	60 (60.00)		

Extrapancreatic organ involvement					
Yes	62	38 (45.16)	24 (54.84)	51.223	<0.001
None	44	4 (31.82)	40 (68.18)		

**Table 5:** Multivariate analysis of recurrence in patients with type I AIP after corticosteroid therapy.

Factors	*β*	SE	Wald *χ*^2^	OR	*P*	95% CI

The time of hormone therapy is short	0.557	0.212	6.903	1.745	0.008	1.152∼2.645
Extrapancreatic organ involvement	0.631	0.145	18.938	1.879	<0.001	1.415∼2.497

Note: *β* (the unstandardized beta (*B*)) represents the slope of the line between the predictor variable and the dependent variable, SE – standard error, OR – odds ratio, and 95% CI – 95% confidence interval).

## Data Availability

The data sets used and analyzed during the current study are available from the corresponding author upon reasonable request.
